The article "A systematic and theoretical approach to the marketing of higher education" was published in 2022. Journal: Front Psychol.

# A systematic and theoretical approach to the marketing of higher education

**DOI:** 10.3389/fpsyg.2022.982347

**Published:** 2022-10-12

**Authors:** Edna Rabenu, Or Shkoler

**Affiliations:** ^1^Tel-Hai College, Tel Hai, Israel; ^2^HEC Montréal, Université de Montréal, Montreal, QC, Canada

**Keywords:** Facet theory, mapping sentence, higher education, marketing, international students, conceptual paper

## Abstract

The aim of this article was to open a hatch to the consumer psychology research through the eyes of Facet Theory. The Facet Theory enables to delve into a concept or an issue under investigation and define it formally, systematically, and comprehensively, but still parsimoniously. In order to better explain its philosophical basis and the principles of this theory, we apply and demonstrate it on the domain of marketing of higher education to students. There are four distinct facets identified in this regard, namely, (A) Achieving Personal Goals, (B) Institution’s Marketing Orientation, (C) Secondary Decision Criteria, and (D) Level of Education. Based on those facets and their related respective elements, a suggested definitional directive for the marketing of higher education to students is construed.

## Theoretical background

In the current paper, a systematic theoretical approach with an immense potential to guide both quantitative and qualitative research paradigms, namely, the Facet Theory, will be presented. It paves a way in which scholars may formulate and/or probe theories, constructs, and philosophical perspectives by interweaving ideas with reality, terminologies, data/information, phenomenologies, ontologies, mereologies, and epistemologies (e.g., Shye, 1991; Hackett, 2018a). Further, it can be applied in any field of knowledge from education (e.g., Friedman, 2008; Fisher, 2016, 2018; Alt, 2018), psychology (e.g., Rabenu et al., 2015; Rabenu and Tziner, 2016; Hackett, 2019), management and organizational behavior (e.g., Shkoler et al., 2017b), to even birds’ behavior (Hackett et al., 2019). The Facet Theory (FT) is limited to neither a specific research paradigm (quantitative vs. qualitative, case studies, etc.) nor a certain knowledge domain, and it can be applied to any. The essence of the Facet Theory analytical approach is funneled into a conceptual entity called a mapping sentence; it offers a meticulous, systematic, and parsimonious definitional framework of any phenomenon under investigation. The current paper focuses on the mapping sentence, giving an exemplary demonstration. Both, the Facet Theory and the mapping sentence, will be elaborated further.

The article is structured as follows: (1) the context of higher education is presented, followed by (2) an explanation about the Facet Theory and the mapping sentence, and finalized with (3) the formulation of a mapping sentence—demonstrated on the marketing of higher education to students. Notably, the paper and the mapping sentence touch the broad domain of higher education and students. However, due to great variability, sensitivity, and complexity within this field, in order to encapsulate all of them, the FT is the prime candidate for the job. To emphasize, the theoretical background relies on the literature of *international students^1^* as their special situation can reflect all students (domestic included), but not vice versa. For instance, in addition to other things, international students also deal with citizenship and residency issues, legal and visa problems, long-distance transportation, unique psychological challenges (e.g., loneliness and discrimination), etc.; these will also be elaborated further, specifically in mapping sentence section. Importantly, consumer psychology harbors marketing as a knowledge field, as the former is multidisciplinary, naturally extending itself *via*: (1) sociology, (2) psychology, (3) social–psychology, (4) economics and marketing, and (5) anthropology (Loudon and Della Bitta, 1993; Chen, 2008; Kotler and Armstrong, 2014; Kotler and Keller, 2016; Jansson-Boyd, 2019; Rabenu and Shkoler, 2020b). This highlights the complexity of the field and promotes the use of the Facet Theory as an indispensable tool to simplify, but formally define, that field.

The article "A systematic and theoretical approach to the marketing of higher education" was published in 2022. Journal: Front Psychol.

## Marketing of higher education

Higher education is often considered a marketable service (e.g., Shkoler and Rabenu, 2020b). Therefore, marketing higher education to students falls under the umbrella domain of consumer psychology (see Hackett, 2018b; Shkoler and Rabenu, 2020b). To elaborate, the decision-making process to “purchase” higher education by students necessitates complex psychological and cognitive processes. Academic institutions need to understand these processes, and by using intelligent marketing to attract prospective students, they can influence their decision making and tilt or support their choices accordingly (Shkoler and Rabenu, 2020b).

Knight (2011), for example, contemplated that education is regarded as a tradable service, birthing new commercial possibilities in cross-border education. On top of that, recruiting (international) students can be considered as a “key migration industry” (Beech, 2018, p. 622).

Marketing higher education to students is challenging as it involves a complex arena with many actors/players: (1) the students; (2) academic institutions; (3) governments; (4) the economic systems (globally and locally); and more (see Beine et al., 2014; Beech, 2018). In this paper, there is a focus on two of the above:

*The students* are the potential *consumers/customers* of higher education, which is why it is of paramount importance to understand their motivations, needs, and expectations (e.g., Prugsamatz et al., 2006; Bunce et al., 2017; Nafari et al., 2017; Shkoler and Rabenu, 2022). By identifying their expectations, meeting them, or even exceeding them altogether, this has the potential to support marketing efforts of higher education institutions (e.g., Prugsamatz et al., 2006; Woodall et al., 2014; Nixon et al., 2018), inducing and increasing customer value (e.g., Chen, 2008).

The article "A systematic and theoretical approach to the marketing of higher education" was published in 2022. Journal: Front Psychol.

*The academic institutions* are the *providers* of higher education, with exceedingly increasing competition among them (Beech, 2018, p. 622). There are several reasons for these institutions (as well as countries) to be courting students, in general, and international students, in particular: tuition fees (as an income source), support for research, potential skilled/talented workers in future, diversity (e.g., cultural and demographical), networks, and more (for further reading, see Shkoler and Rabenu, 2022). As such, these academic institutions must be aware of and try to actively discover prospective students’ needs, motivations, preferences, and wants (see Appendix 2 in Shkoler and Rabenu, 2022), resulting in the application of the prospective student to the institution, in order to ensure sustainable higher education.

## Facet theory

Research, particularly in the social sciences, usually involves complex phenomena, variables, and processes (e.g., Friedman, 2008; Tziner, 2018; Roazzi and Souza, 2019). To illustrate, it is not trivial to understand and define complex concepts such as values, intelligence, motivation, and attitudes. While striving to achieve high-quality research and in order to conceptualize these concepts, we need to expose their intricate components and their interrelationships. It is obvious that poor conceptual definition of content domains impinges the generation and accumulation of knowledge and impairs, for example, the replicability of research (Tziner, 2018).

In this article, we suggest using Facet Theory as a venerable and systematic paradigm for conceptualizing complex phenomena (e.g., Shkoler et al., 2017b). As a demonstrative example, an application of this theory is done on the marketing of higher education to students.

The Facet Theory is a method that facilitates and fosters formal definitions of components of a problem or the issue under investigation (Guttman, 1957), and hence, it allows for the depiction of a complex interplay of variables (Guttman and Greenbaum, 1998; Hackett, 2014; Roazzi and Souza, 2019; Solomon(Ed.)., 2021). In FT, the universe of observations is formally defined. Additionally, FT weaves this by testing hypotheses (about the relationship between the definitional framework and the structure of the empirically oriented observations) (Elizur, 1984). To elaborate, FT provides both the definitional system of the universe of observations and the rationale for hypotheses of a research both quantitative (Levy, 1985; For further reading, see Guttman and Greenbaum, 1998; Roazzi and Souza, 2019; Solomon(Ed.)., 2021) and qualitative (e.g., Hackett, 2016, 2021a). However, FT has invaluable contribution to the definition of concepts, based on using mapping sentence as the definitional framework, regardless of whether it is applied in followed-up quantitative research or not (e.g., Schlesinger, 1991; Hackett, 2016, see ahead). In any case, adopting the FT entails that the researcher will most probably jungle multiple variables simultaneously, that is—until the creation of their combined formulation into harmonious and meaningful declaration of the domain of research. However, utilizing FT can be challenging and quite uncommon (Hackett, 2021a, p. X).

The article "A systematic and theoretical approach to the marketing of higher education" was published in 2022. Journal: Front Psychol.

Simply put, a *facet* is articulated as a group of common characteristics/traits, and this group represents semantic components of a desired context field (Yaniv, 2011). More specifically, a facet is “a classification of item domains of a given content universe according to some rule” (Elizur, 1984, p. 380). These common traits are dubbed as *elements* (of a facet). A set of finely defined facets (and their respective elements) comprise the essence of FT—the mapping sentence.

## Definitional framework and the mapping sentence

The definitional framework for formally defining a content universe is called a “mapping sentence.” It is the basic tool offered by the FT (e.g., Guttman, 1957; Canter, 1985; Borg and Shye, 1995). It serves as a guide and a beacon for: (1) first formulating hypotheses; then (2) creating structured assumptions; then (3) constructing systematic measures; then (4) planning and collecting observations; and finally (5) analyzing the data (e.g., Levy, 2005); it is the heart of the FT approach (Hackett, 2014, p. 67).

Moreover, after to Levy (1985, p. 60), a mapping sentence, which defines a universe of observations for a selected theory, has the following three main components: (1) the target population (to be classified), (2) the spectrum of variables (constituting the criteria for the classifications), and (3) the category range for each variable (see also Shye, 1991). The mapping sentence includes these three kinds of sets. It combines several exclusive *facets* (categories that classify variables under a specific and unifying rule), which define the content universe of the domain or area of the study. Every facet may contain multiple *elements* (“sub-categories”), with a minimum of two elements per facet, which also must fit the facet’s rule. The facets are connected between them by text, while all are delineated by a common range (e.g., Elizur, 1984; Shye, 1991; Tziner, 2018). By way of illustration, a mapping sentence “looks” and reads like an ordinary sentence.

The article "A systematic and theoretical approach to the marketing of higher education" was published in 2022. Journal: Front Psychol.

In essence, there are two kinds of mapping sentences, namely, *empirical* (also named “general”) *and theoretical* (also named “declarative”) (Schlesinger, 1991; Hackett, 2016, 2021a). More specifically, empirical mapping sentence may lead to the creation of a research measure (operationalization) and research hypotheses followed by either support or falsifying of hypotheses (see, e.g., parental involvement perception by Fisher, 2016; (re)defining workaholism by Shkoler et al., 2017b; and defining coping with stress by Rabenu et al., 2015).

With regard to the theoretical mapping sentence, however, Hackett (2016, 2021a) argues for the utility of use of the mapping sentence as a standalone philosophically coherent approach when attempting to understand the phenomenological human experience. Further, he perceived mapping sentence as a tool to investigate the hermeneutical consistency of research, forming a precise, though flexible, framework in philosophical and qualitative psychological research (Hackett, 2016, p. 5; see also Schlesinger, 1991). This mapping sentence can lead to the definition of very complex concepts without necessitating a follow-up empirical research (see, e.g., Rabenu and Tziner, 2016—defining resilience; Rabenu and Hackett, 2017—defining work discrimination).

It is important to emphasize that one of the main contributions and properties of the mapping sentence, by and large, is its ability to provide a comprehensive definition of a phenomenon, in a parsimonious manner (e.g., Shkoler et al., 2017b). For further reading, we recommend reading Hackett (2018a) and Tziner (2018).

Of note, in this article the focus is on a theoretical mapping sentence in the qualitative sense; the declarative mapping sentence will be elaborated on further. Hackett (2016, 2018a, 2019, 2021a,b) defined the declarative mapping sentence (DMS), as “…a specification of the research domain of interest in terms of the domain’s important components that have appeared in the literature along with the sub-types or elements of each facet, joined in a sensical manner to express a hypothesis regarding the experiential nature of the research domain” (Hackett, 2021b, p. 2). Therefore, from a qualitative point of view, the DMS is a proposition that serves as a solid surface for developing research instruments to gather information (up-bottom). However, the DMS can also serve researchers in the opposite direction, namely, bottom-up. In this case, such as in the grounded theory approach (Glaser and Strauss, 1967), the researchers document what happens in the field, analyze the collected data, and may use the DMS as a tool for systematic thinking which will assist them in building their theoretical background and arguments, while the facets serve as themes themselves (Hackett, 2021b). Also, as opposed to the *empirical* mapping sentence, the DMS need not include the commonly used “range facet,” but rather ends in a qualitative outcome (by the declarative nature of the mapping sentence) (Hackett, 2021a,b,c).

The article "A systematic and theoretical approach to the marketing of higher education" was published in 2022. Journal: Front Psychol.

In this article, we construct and present a theoretical mapping sentence that we believe represents the content of the marketing higher education to students, for the goal of demonstrating the DMS is the exemplary demonstration in the current article as this issue includes, *inter alia*, subjective experience and perceptions of the prospective students which better fit the qualitative research approach, both phenomenologically and epistemologically; qualitative research explores phenomena that are difficult to quantify by measurement or mathematics (e.g., beliefs, experiences, and knowledge) (Brod et al., 2014).

## Formulating the mapping sentence

We capitalize on vast literature of the drivers and reasons that individuals seek higher education internationally (Facet A), different marketing approaches (e.g., the 4Ps; Borden, 1964; McCarthy, 1964. For further reading, see Kotler, 1999) that academic institutions may use to suit their needs (Facet B), understanding of the plethora of constraints that these students need to cope with (Facet C), in tandem with the level of education pursued (Facet D). As such, one of the main goals of the current paper was to offer a systematic theoretical framework for marketing higher education to students (as mentioned in “Theoretical Background” section, the examples and content broadly touch students, but specifically on international prospectives). To this end, we utilize the Facet Theory analytical approach to formulate a comprehensive yet parsimonious mapping sentence (i.e., systematic definition), as directions for higher education institutions and marketing personnel. The suggested formulated mapping sentence is depicted in Figure 1, and each of its components is elaborated further.

**FIGURE 1:** Mapping sentence of marketing higher education to students.

The article "A systematic and theoretical approach to the marketing of higher education" was published in 2022. Journal: Front Psychol.

## Facet A: Achieving personal goals

As opposed to regular travelers or tourists, international students *actively pursue* higher education abroad (e.g., King and Gardiner, 2015). Notwithstanding, these students seek higher education for three main reasons, but, ultimately, all of them revolve around enhancing the concept of the self and in other words enhancing the (1) human capital, (2) financial capital, and/or (3) psychological capital.

### Element a1: Human capital

This is the knowledge, skills, and abilities of an individual, usually measured by the (highest) level of education and by the practical “know-how” experience (e.g., Luthans and Youssef, 2004; Luthans et al., 2004; Felício et al., 2014). Prospective students often seek out “the best” education possible for them, and sometimes, this can only be found in foreign countries (Findlay et al., 2012). Thus, acquiring higher(est) levels of education is a venerable approach to increase one’s human capital (e.g., Bourdieu, 1986; Findlay et al., 2012), as it may be a “distinguishing identity marker” (Findlay et al., 2012, p. 128; Lomer et al., 2018; e.g., higher social status, prestige, and reputation; Bourdieu, 1986). Lastly, as this is active (i.e., by choice) enhancement of human capital, there is another aspect to that—passive (i.e., absorption) enhancement—for example, by learning a new language or culture in the destination country (e.g., Cubillo et al., 2006; Yang, 2007; Varghese, 2008; Hyams-Ssekasi et al., 2014; Tan, 2015; Wu et al., 2015; Lewis, 2016; Nathan, 2017; Huong and Cong, 2018).

### Element a2: Financial capital

Evidently, individuals with higher/better education often earn higher wages in return and, hence, experience less unemployment (Card, 1999, p. 1802. See also Becker, 1964). In essence and economic terms, there is a consideration of costs–benefits when individuals decide to migrate abroad (González et al., 2011), and international students often seek to increase their employability and financial status in future (Beine et al., 2014; Huong and Cong, 2018) and have more career opportunities (Cubillo et al., 2006; Yang, 2007; Lewis, 2016).

### Element a3: Psychological capital

It is defined as a positive psychological state of an individual characterized by: self-efficacy, optimism, hope, resilience, gratitude, flow, courage, creativity, forgiveness, authenticity, emotional intelligence, and more (Luthans et al., 2015). It “involves investing in the actual self to reap the return of becoming a possible self” (Avolio and Luthans, 2006, p. 147; see also Luthans et al., 2004). Hence, prospective students believe that it is possible to develop and augment this capital *via* higher education in a foreign country (as previously mentioned, this is usually considered as superior to obtaining this kind of capital in their home country). They seek, therefore, psychological growth (Yakunina et al., 2013) through improving their: self-efficacy, independence, personal pride, acceptance of ambiguity, experience of a different culture or even teaching methods, discovering new places, etc., (e.g., Mazzarol and Soutar, 2002; Cubillo et al., 2006; Yang, 2007; Varghese, 2008; Jianvittayakit and Dimanche, 2010; Tan, 2015; Lewis, 2016; Nathan, 2017; Huong and Cong, 2018). Lastly, it is important to note that hedonistic desires are a part of the psychological capital (i.e., pleasure fulfillment and sensuous gratification; Schwartz, 2012). Meaning, students choose to study abroad also for reasons such as traveling opportunities, liberal sex, local drinking culture, and living without (m)any commitments (e.g., Yang, 2007; Jianvittayakit and Dimanche, 2010; Nghia, 2015; Lewis, 2016; Nathan, 2017; Huong and Cong, 2018).

The article "A systematic and theoretical approach to the marketing of higher education" was published in 2022. Journal: Front Psychol.

## Facet B: Institution’s marketing orientation

Regardless of what motivation is driving the prospective students, higher education institutions worldwide have different marketing strategies, education offered, and competitive advantages. As such, approaching a prospective student can be delicate, as they seek different things, and the institution will need to (re)consider its marketing and branding positions(e.g., Ivy, 2008; Khilukha et al., 2020; Lim et al., 2020). Commonly used in a marketing mix, the 4Ps model remains very prominent (Borden, 1964; McCarthy, 1964; see also Kotler, 1999) and entails the following four main marketing foci (approaches): (1) price, (2) product, (3) place, and (4) promotion.

### Element b1: Price

It is defined as everything (tangible/intangible) given by the buyer/acquirer (in terms of money, time, and effort given) to obtain a product; it tackles the *customer cost* aspect of the exchange (Kotler, 1999; Yudelson, 1999). For higher education, an institution (university/college) wishing to position itself in this approach may want to emphasize the benefits it offers regarding the charged fees for enrollment (e.g., tuition fees, flexibility in paying them, flexibility of the tuition approach, etc.) (Ivy, 2008; Lim et al., 2020).

### Element b2: Product

It is defined as the clear benefits the user will obtain from the purchase/exchange through time; it tackles the *customer solution* aspect of the exchange (Kotler, 1999; Yudelson, 1999). For higher education, an institution may wish to emphasize, for example, aspects related to the curriculum of the degrees and diplomas it offers (e.g., range of choice of majors and electives). Additionally, the institution can highlight other incentives which may add special value to the degree (e.g., total number of credits for the degree, availability of on-campus accommodation, exchange opportunities for international students, students’ racial diversity, more liberal environments, residential requirements of the diploma/degree, the size of classes, etc.). In addition, the image of the university/college can also be capitalized on (e.g., academic reputation of the faculty/staff, institution’s reputation *via* press reviews and leading league tables, the online website’s content, and sophistication of the institution in demonstrating the reputation of each of its schools, prestige, status, and more) (Ivy, 2008; Lim et al., 2020).

The article "A systematic and theoretical approach to the marketing of higher education" was published in 2022. Journal: Front Psychol.

### Element b3: Place

It is defined as the consideration of where the product is made available and how it is, *de facto*, displayed; it tackles the *convenience* aspect of the exchange (Kotler, 1999; Yudelson, 1999). For higher education, an institution may wish to emphasize the attractiveness of the place it is situated in (e.g., a “cool” city, a lavish country, proximity to public transportation and ease of transit, availability of shuttles to the institution, traveling/touristic opportunities, liberal culture, proximity to nature/vistas, can registration be made online in addition to on-site? is information about the programs made available online? etc.) [for further reading, see Rabenu and Shkoler (2020a)].

### Element b4: Promotion

It is defined as all of the information transmitted among parties in the exchange/purchase, and the *communication*, of the exchange, to the consumers that they “need” this specific product (Kotler, 1999; Yudelson, 1999). For higher education, an institution may wish to employ standard mass advertising, done through the traditional media for the communication of the information about its brand, offerings, degrees, and other important aspects of the product—to target markets (e.g., publicity and public relations, press advertising, electronic and online media, etc.) (Ivy, 2008; Lim et al., 2020).

## Facet C: Secondary decision criteria

Motivation alone (i.e., Facet A) is usually an insufficient drive force. There are secondary decision criteria that may either push or hamper (support and enhance vs. constrain and inhibit) the prospective student toward their final decision to study abroad. There are quite several such conditioning/moderating [e.g., Appendix in Shkoler et al. (2017a)] factors, each with a different effect and impact on the decision: (1) formal/legal requirements, (2) social resources, (3) psychological resources, (4) financial reserves, (5) demographical status, (6) transportation accessibility, (7) home–destination countries’ affiliations/ties, (8) language familiarities/barriers, and (9) recommendations or criticisms. Each element will be elaborated succinctly: when favorable—they will support the decision; when not—they will inhibit it.

The article "A systematic and theoretical approach to the marketing of higher education" was published in 2022. Journal: Front Psychol.

### Element c1: Formal/legal requirements

Examples are higher education difficulties at home [such as fees, admission and difficulty of gaining entry, and (un)availability of programs]; impact of legal procedures in the destination country (such as immigration, legislation, and visa); and facilitated admissions in the destination institute (such as recognition of previous qualifications, certificates and/or diplomas, and easier processes) (e.g., Becker and Kolster, 2012; Ahmad et al., 2016; Huong and Cong, 2018).

### Element c2: Social resources

Social networks and relationships are in either the home or destination countries that can potentially provide financial, emotional, and/or physical support for the prospective student, such as family or friends (Mazzarol and Soutar, 2002; Li and Bray, 2007; Yang, 2007; Becker and Kolster, 2012; Beine et al., 2014; Nghia, 2015; Tan, 2015; Lewis, 2016; Tantivorakulchai, 2018).

### Element c3: Psychological resources

Relocating to another country is usually accompanied with varying levels of uncertainty, challenges, and difficulties (e.g., hostility, bias, stress, loneliness, and more; Sawir et al., 2008; Rienties and Nolan, 2014; Lee, 2015; Poyrazli, 2015; Yan and Pei, 2018). Personal characteristics (e.g., self-efficacy and resilience) that can support the migration are essential for a better assimilation in the destination country, stress coping, and adaptation (Kosic et al., 2004; Chen, 2007, 2008; Wang, 2009; Ramelli et al., 2013; Yakunina et al., 2013; Mak et al., 2015; Meshulam and Harpaz, 2015; Kashima et al., 2017).

### Element c4: Financial reserves

International higher education is often expensive (Rabenu and Shkoler, 2020a). Tuition fees, other studying costs, and living costs impinge the capacity for self-sustenance, and, therefore, the monetary reserves one has can definitely aid in relocating (e.g., Becker and Kolster, 2012; Beine et al., 2014; Lewis, 2016; Huong and Cong, 2018).

### Element c5: Demographical status

Simply put, the marital and sociodemographic status of the prospective student may have profound impacts on the decision to relocate (e.g., parenthood, marriage, etc.; Baldridge et al., 2006). Relocating an entire household is much more difficult than migrating on one’s own, both logistically and bureaucratically.

The article "A systematic and theoretical approach to the marketing of higher education" was published in 2022. Journal: Front Psychol.

### Element c6: Transportation accessibility

Nowadays, various transportation modes and widespread routes have improved the accessibility to universities and colleges around the world (Lee, 2015). Additionally, this is based on the: (1) *availability* of transportation inside and/or between countries; (2) *costs* of the transportation; and (3) importance of the *geographical proximity* between home and destination countries (e.g., Becker and Kolster, 2012; Beine et al., 2014; Tan, 2015; Ahmad et al., 2016; Huong and Cong, 2018).

### Element c7: Affiliations/ties between home and destination countries

The relationship between countries is an important aspect in relocating. Sharing sociohistorical and cultural similarities can encourage students to migrate from their home country to another country boasting similar characteristics (e.g., Argentinians and Colombians moving to Spain; Lasanowski, 2011). This is based on many considerations, such as religious, economic, political, linguistic, cultural, historical, and colonial (e.g., Cubillo et al., 2006; Bolsmann and Miller, 2008; Varghese, 2008; Kishun, 2011; Becker and Kolster, 2012; Nathan, 2017; Huong and Cong, 2018).

### Element c8: Language familiarities/barriers

Language has a cardinal role as a key mobility motivator (Misra et al., 2003; Andrade, 2006; Lasanowski, 2011). Language barriers, on the contrary, also hamper learning, communication, understanding of academic tasks and assessments, and technical necessary language (e.g., in laws, psychology, business administration, marketing, and more) and, ultimately, may impair academic writing and achievements (Andrade, 2006; Cubillo et al., 2006; Yang, 2007; Varghese, 2008; Wilkins et al., 2012; Beine et al., 2014; Wu et al., 2015; Lewis, 2016; Cowley and Hyams-Ssekasi, 2018).

### Element c9: Recommendations or criticisms

Trustworthy significant others and other sources (e.g., family, agents, sponsors, friends and peers, ex-students, professors and teachers, etc.) can support or impinge on a decision to study abroad by either giving a recommendation or providing criticisms (Mazzarol and Soutar, 2002; Cubillo et al., 2006; Maringe and Carter, 2007; Hildén, 2011; Jon et al., 2014; Huong and Cong, 2018; Santos et al., 2018). Notably, personal experience (e.g., alumni) is perceived to be highly trustworthy and is held in greater regard than random suggestions.

## Facet D: Level of education

Beyond basic motivation (i.e., Facet A), the level of education, that is the degree sought after, is, by definition, an integral and axial part of the decision to study abroad. To illustrate, graduate students (pursuing a *research* degree) usually differ from other students (seeking a *professional* degree) and from *undergraduates*. For example, Mpinganjira (2009) has found that *undergraduates* were driven by seeking more experience and career opportunities. On the contrary, *postgraduate* students were (de)motivated by the (un)availability of courses at their home country (notably, neither group was affected by the entry and/or admission technicalities). Furthermore, graduates seek to acquire higher education internationally for the purpose of gaining higher-quality education (Kim et al., 2018). As such, three main education levels are critical in deciding how to market higher education to international students, as in each case, the baseline motivations, incentives, and drives to choose a certain program (and where) are quite different from one another: (1) undergraduate, (2) graduate, and (3) postgraduate.

The article "A systematic and theoretical approach to the marketing of higher education" was published in 2022. Journal: Front Psychol.

### Element d1: Undergraduate

Seek to acquire an undergraduate (bachelor’s, B.A.) degree.

### Element d2: Graduate

Seek to acquire a graduate (master’s, M.A.) degree.

### Element d3: Postgraduate

Seek to acquire a postgraduate (doctorate, Ph.D.) degree.

These were the concrete and substantive facets, which leave a common outlining facet to be introduced—the range facet.

## Discussion

The current article had two main goals. The first is to present the Facet Theory as a recommended methodology when defining concepts (new or otherwise) in a systematic and comprehensive manner. This is done with the utilization of the mapping sentence as the directive of the definition, and one of the main tools FT offers the researcher. The second is to demonstrate an application of the FT *via* a definition to a specific domain—marketing higher education to students. As was illustrated and elaborated, the (theoretical/declarative) MS allowed for setting an organized (formally and systematically) and well-planned definition that encompasses the comprehensive content world in the specific domain previously mentioned. This definition may be used in follow-up research in construction of qualitative tools and methods that will rely on the MS, in order to collect information from the informants—prospective student candidates. On the contrary, qualitative researchers who have already collected these data from students about their experience with the marketing of higher education programs are encouraged to use the MS in this article as a solid theoretical basis to their thematic analysis when the facets are used as themes.

## Limitations

The literature is aware, however, that there are researchers who might view the systematic and methodic framing of the MS as rendering the phenomenological richness as superficial and shallow. Nevertheless, the rich description of feelings and lived experiences that may arise from any research field does not contradict the MS, but can build, support, or use it (Shye, 1991).

The article "A systematic and theoretical approach to the marketing of higher education" was published in 2022. Journal: Front Psychol.

In addition, we stress that the MS in the current paper is conditioned by the culture of the prospective student just as well as by the culture of the academic institutions (i.e., different cultures exhibit distinguished needs, motivations, aspirations, and wants; e.g., human capital, etc.). Because we used “Western point of view,” the generalizability of the MS is somewhat diminished.

Lastly, the current MS was construed without consultation with experts in the field, thus reducing its content validity^2^. Traditionally, exploring such validity is qualitative in nature (Hinton and Platt, 2018). To elaborate, the researcher ought to approach around 5–10 subject matter experts (SMEs)—individuals within the relevant field, versed in the relevant practitioner and/or academic knowledge (see, e.g., Hinton and Platt, 2018, p. 71). These experts are, for example, marketing managers, academic program managers, student services administration, researchers in higher education and education management, and others. These experts are tasked with (1) making judgment to the degree to which each individual element in the MS is relevant and content-valid to the framework of the MS itself (i.e., marketing higher education to students) and (2) evaluating the MS in its entirety, as a whole entity (see Brod et al., 2014; Hinton and Platt, 2018). These methods are reactive in essence, and as such, we also suggest a more proactive approach to establishing content validity in this regard. It would be very beneficial to create a workshop in which SMEs will be educated in brief in the FT and, specifically, on how to construct and design an MS. Following this, they will be asked to generate an MS, and then, we will assess and compare the alignment and convergency of their MS and ours, making necessary adaptations and amendments as required.

## Future recommendations

Although the current paper was philosophical and qualitative in nature, due to the complexity of the field (i.e., consumer psychology and marketing) it is encouraged to use a mixed-method research approach to unveil “more sides of the same coin” (e.g., Shkoler, 2018); both methods may synergize to produce a more refined mapping sentence and a better understanding of the field.

The MS (Figure 1) can be used as a compass and directive for academic institutions to compile their own marketing mix to attract students to their ranks. To this end, academic institutions may design a survey that is based on the different elements comprising the MS (Figure 1), thus helping them by better understanding the students’ motivations, experiences, expectations, needs, and aspirations. An example for such a tool which focuses on the motivations of students, particularly, can be seen in Shkoler and Rabenu (2022). Example items from the Initial/Basic Prospective (International) Students Needs Survey include: (1) for Facet A (Achieving Personal Goals): “I am interested in achieving personal goals, to increase my **human** capital (such as knowledge and skills): _____” or “I am interested in achieving personal goals, to increase my **psychological** capital (such as self-confidence and resilience): _____”; (2) for Facet C (Secondary Decision Criteria): “The extent of your social resources (such as family, friends, and acquaintances): _____” or “Language barriers or familiarity (the extent of familiarity with the local language in speech, reading and writing): _____.” For further reading, see Appendix 2 in Shkoler and Rabenu (2022).

The article "A systematic and theoretical approach to the marketing of higher education" was published in 2022. Journal: Front Psychol.

The current paper is of a basic research design and is conceptual in essence, based on purely academic literature. It is philosophical and not applied. As such, it is highly recommended to confirm the MS’s viability and credibility by subject matter experts and/or relevant personnel (see also “Limitations” section). All in all, based on the MS, we may suggest few channels for applied actions that can be either specific or generic and can be taken in most institutions, for example (1) using digital marketing in social media to increase informal ranking of the institution (e.g., element c9); (2) raising awareness in the marketing departments for the complexity and sensitivity surrounding marketing higher education to students in the increasingly competitive academic world; (3) gauging the effectiveness of current marketing mix and actions to attract students, making changes as required; (4) monitoring student retention post factum according to specific criteria (e.g., based on Facet C in the MS; Figure 1); and more.

## Data availability statement

The original contributions presented in the study are included in the article/supplementary material, further inquiries can be directed to the corresponding author/s.

## Author contributions

ER: conceptualization, writing, original draft, and reviewing and editing. OS: writing, reviewing, editing, and visualization. Both authors approved the manuscript for publication.

## Footnotes

1 An international student is defined as “an individual whose primary goal is the acquisition of (some form of) higher education in a country in which he or she has *no* permanent residential status and *no* local citizenship, regardless of the studying method” (Shkoler and Rabenu, 2020a, p. 19).

2 *Content validity*: “derived during concept elicitation, is the measurement property that assesses whether items are comprehensive and adequately reflect the… perspective for the population of interest” (Brod et al., 2014, p. 5257) and it is “a measure of the degree to which the items within a scale *appear* to measure the construct of interest, as judged by subject matter experts” (Hinton and Platt, 2018, p. 61; italics are in the original article).
